This article has been retracted.

# Emphysematous Cystitis: A Radiological Diagnosis of Potentially Life-Threatening Infection

**DOI:** 10.7759/cureus.20201

**Published:** 2021-12-06

**Authors:** Shouq A Alhusayni, Thekra H Alshammari, Abdullah A Althomali, Mishari M Alqahtani, Waad A Alanazi, Mohammed A Alghamdi, Faisal M AlDawsari, Elan M Homoud, Abdulrahman A Alharbi, Khalid E Althobaiti, Abdulrahman A Alsubaihi, Abdullah M Alsayed, Abdalmohsen M Albaqami, Ahmad M Alamer, Faisal Al-Hawaj

**Affiliations:** 1 College of Medicine, University of Hail, Hail, SAU; 2 College of Medicine, Taif University, Taif, SAU; 3 Family Medicine, Prince Sultan Military Medical City, Riyadh, SAU; 4 College of Medicine, Northern Border University, Arar, SAU; 5 College of Medicine, Medical University of Lodz, Lodz, POL; 6 College of Medicine, Majmaah University, Al Majma'ah, SAU; 7 College of Medicine, King Saud Bin Abdulaziz University for Health Sciences, Riyadh, SAU; 8 College of Medicine, King Abdulaziz University, Jeddah, SAU; 9 College of Medicine, Arabian Gulf University, Manama, BHR; 10 College of Medicine, Imam Abdulrahman Bin Faisal University, Dammam, SAU

**Keywords:** computed tomography, case report, abdominal pain, emphysematous, urinary tract infection, cystitis

## Abstract

Urinary tract infections are very prevalent among women. The majority of urinary tract infections are uncomplicated and can be managed empirically with no further investigations. However, imaging studies may be indicated in patients with severe or persistent symptoms. Complicated urinary tract infections typically develop in the setting of diabetes mellitus. We report a case of a 52-year-old woman who presented to the emergency department with severe lower abdominal pain for two days that was associated with nausea, vomiting, and fever. There was no history of change in urine or bowel habits. Besides the history of well-controlled asthma, the patient was not known to have any comorbid medical condition. Upon examination, the patient had tachycardia, low-grade fever, and a localized suprapubic tenderness with guarding. Laboratory investigation revealed leukocytosis, elevated erythrocyte sedimentation rate and C-reactive protein, and deranged renal functions. Further, urinalysis revealed numerous white blood cells, red blood cells, positive nitrite, and leukocyte esterase. A computed tomography scan demonstrated the presence of small locules of gas within the lumen and the wall of the bladder representing emphysematous cystitis. The patient was admitted to the intensive care unit. She received aggressive hydration therapy and a short course of opioid therapy for pain control. Broad-spectrum antibiotic therapy in the form of piperacillin-tazobactam was initiated. Over the following few days, the patient exhibited significant improvement in his symptoms and resolution of the laboratory parameters. Emphysematous cystitis is a rare infection of the lower urinary tract with gas formation. The case highlighted that such a condition may develop in the absence of diabetes mellitus or other risk factors. Prompt treatment is crucial as emphysematous cystitis can be life-threatening if the diagnosis is missed or delayed.

## Introduction

Urinary tract infections, including cystitis and pyelonephritis, are extremely prevalent among women. As women have a shorter urethra, this explains why they have a higher tendency to develop urinary tract infections. The diagnosis of urinary tract infection is based on the clinical signs and symptoms. Indeed, the likelihood of having cystitis exceeds 90% in women with urinary frequency and dysuria without vaginal discharge [1]. Hence, simple cystitis can be managed empirically without the need for further investigations. The diagnosis of simple cystitis, however, should exclude the presence of signs of systemic disease, including fever, chills, and rigors. Imaging studies are indicated for patients with persistent symptoms despite receiving the appropriate therapy, severe symptoms suggestive of sepsis, or renal function tests suggestive of urinary obstruction [2]. Imaging aims to exclude obstruction or complication such as abscess formation that delays the response to therapy. Here, we present a case of a middle-aged woman with severe lower abdominal pain who was diagnosed as having emphysematous cystitis. It is worth noting that she did not have any risk factor for this severe infection, which is very unusual in patients with emphysematous cystitis [3].

## Case presentation

We present a case of a 52-year-old woman who presented to the emergency department with severe lower abdominal pain for two days. The pain was non-radiating, constant, progressing in severity, and stabbing in nature. She scored the pain as 7 out of 10 on the severity scale. The pain was not related to urination, meal intake, or posture. She attempted over-the-counter analgesics but they did not result in any improvement. The patient also complained of fever and nausea, and had one episode of vomiting. There was no change in urine or bowel habits.

Besides the history of well-controlled asthma, the patient was not known to have any comorbid medical condition. She underwent laparoscopic cholecystectomy for recurrent attacks of biliary colic. Her medications included inhaled corticosteroids for asthma and nutritional supplements. She had no history of allergies to food or drugs. The patient was a smoker of 15 packs a year and had no history of alcohol consumption. She worked as an accountant. The family history was remarkable for sickle cell disease.

Upon examination, the patient appeared in distress because of the pain. Her vital signs revealed tachycardia (114 bpm), low-grade fever (37.9℃), normal respiratory rate (15 bpm), and maintained blood pressure (114/73 mmHg). The oxygen saturation was maintained on room air. Abdominal examination revealed a localized suprapubic tenderness with guarding. No palpable mass was appreciated. Bowel sounds were normal. Examination of other systems revealed no abnormalities.

Initial laboratory investigation revealed leukocytosis (14,000/μL), elevated erythrocyte sedimentation rate (26 mm/hr), and elevated C-reactive protein (16 mg/dL). The renal profile showed derangement of the urea (25 mg/dL) and creatinine levels (1.4 mg/dL). The hepatic profile was normal (Table 1). Urinalysis revealed numerous white blood cells (>100 cells), red blood cells (>100 cells), and positive nitrite and leukocyte esterase. The urine specimen was taken for culture, which later yielded the growth of *Escherichia coli*.

**Table 1:** Summary of the results of laboratory findings.

Laboratory investigation	Unit	Result	Reference range
Hemoglobin	g/dL	13.7	13.0–18.0
Leukocytes	1000/mL	14.0	4.0–11.0
Platelet	1000/mL	348	140–450
Erythrocyte sedimentation rate	mm/hr.	26	0–20
C-reactive protein	mg/dL	16	0.3–10.0
Total bilirubin	mg/dL	1.2	0.2–1.2
Albumin	g/dL	4.5	3.4–5.0
Alkaline phosphatase	U/L	55	46–116
Gamma-glutamyltransferase	U/L	42	15–85
Alanine transferase	U/L	21	14–63
Aspartate transferase	U/L	17	15–37
Blood urea nitrogen	mg/dL	25	7–18
Creatinine	mg/dL	1.4	0.7–1.3
Sodium	mEq/L	139	136–145
Potassium	mEq/L	3.7	3.5–5.1
Chloride	mEq/L	104	98–107

The patient was administered intravenous lornoxicam for pain control. However, this did not result in a complete resolution of her pain. Subsequently, a computed tomography scan of the abdomen was performed with intravenous contrast. The scan demonstrated the presence of small locules of gas within the lumen and the wall of the bladder. No pneumoperitoneum was noted to suggest perforation. Such radiological findings conferred the diagnosis of emphysematous cystitis (Figure 1).

**Figure 1:** Selected axial (A) and coronal (B) CT images of the lower abdomen demonstrate the presence of gas (arrow) within the bladder wall representing emphysematous cystitis.

The patient was admitted to the intensive care unit. She received aggressive hydration therapy and a short course of opioid therapy for pain control. Broad-spectrum antibiotic therapy in the form of piperacillin-tazobactam was initiated. A transurethral Foley catheter was placed with gravity drainage. Over the following few days, the patient exhibited significant improvement in his symptoms and resolution of the laboratory parameters. She was discharged after 14 days of hospitalizations and five days of stay in the intensive care unit. After 12 months of follow-up, the patient did not have any recurrence or active complaints.

## Discussion

We reported a rare case of emphysematous cystitis in a middle-aged woman with no comorbidities or risk factors. Emphysematous cystitis refers to an infection associated with gas formation. In one of the largest retrospective studies on emphysematous urinary tract infections, Huang and Tseng [4] found that over 95% of patients had diabetes mellitus. Further, a prior study found that urinary obstruction was present in all non-diabetic patients with emphysematous cystitis [5]. In the present case, however, the patient did not have a history of diabetes mellitus and the computed tomography images showed no hydronephrosis or hydroureter to suggest urinary tract obstruction.

The clinical manifestations of emphysematous cystitis are non-specific. Hence, the diagnosis is made based on the imaging studies. As in the present case, an abdominal computed tomography scan reveals the presence of gas in the lumen and the wall of the bladder. While the presence of gas within the bladder wall typically represents emphysematous cystitis, gas within the lumen of the bladder can result from a fistula or following urologic interventions [6]. Emphysematous cystitis typically develops due to infection by *E. coli* or *Klebsiella pneumoniae*. Also, other organisms such as *Proteus*, *Pseudomonas*, and *Candida* can be the causative pathogens [5].

Aggressive medical therapy with appropriate antibiotic therapy is usually sufficient for the treatment of emphysematous cystitis. On rare occasions, the patient may require surgical intervention with bladder debridement or partial cystectomy [7]. However, in the present case, the patient had a significant response to antibiotic therapy and did not require any surgical intervention. Emphysematous cystitis can be life-threatening if the appropriate treatment is not initiated promptly and is reported to have a mortality rate of 7% [8].

## Conclusions

Emphysematous cystitis is a rare infection of the lower urinary tract with gas formation. The case highlighted that such a condition may develop in the absence of diabetes mellitus or other risk factors. Considering its non-specific clinical manifestations, physicians should maintain a high index of suspicion and keep a low threshold for performing cross-sectional studies in patients with severe symptoms and abnormal urinalysis results. Prompt treatment is crucial as emphysematous cystitis can be life-threatening if the diagnosis is missed or delayed.
